# Bone Quantification Around Chitosan-Coated Titanium Dental Implants: A Preliminary Study by Micro-CT Analysis in Jaw of a Canine Model

**DOI:** 10.3389/fbioe.2022.858786

**Published:** 2022-04-07

**Authors:** Nansi López-Valverde, Antonio López-Valverde, Marta Paz Cortés, Cinthia Rodríguez, Bruno Macedo De Sousa, Juan Manuel Aragoneses

**Affiliations:** ^1^ Department of Medicine and Medical Specialties, Faculty of Health Sciences, Universidad Alcalá de Henares, Alcalá de Henares, Spain; ^2^ Department of Surgery, University of Salamanca, Instituto de Investigación Biomédica de Sala-manca (IBSAL), Salamanca, Spain; ^3^ Faculty of Dentistry, Universidad Alfonso X El Sabio, Villanueva de la Cañada, Spain; ^4^ Department of Dentistry, Universidad Federico Henríquez y Carvajal, Santo Domingo, Dominican Republic; ^5^ Institute for Occlusion and Orofacial Pain Faculty of Medicine, University of Coimbra, Polo I‐Edifício Central Rua Larga, Coimbra, Portugal

**Keywords:** titanium dental implant, chitosan-coating, micro-computed tomography, canine model, osteointegration

## Abstract

Surface treatments of Ti in the dental implant industry are performed with the aim of in-creasing its bioactivity and osseointegration capacity. Chitosan (Cht) is a polysaccharide that has been proposed as a promising biomaterial in tissue engineering and bone regeneration, due to its ability to stimulate the recruitment and adhesion of osteogenic progenitor cells. The aim of our preliminary study was to evaluate, by micro-computed tomography (micro-CT), the osseointegration and bone formation around Cht-coated implants and to compare them with conventional surface-etched implants (SLA type). Four im-plants (8.5 mm length × 3.5 mm Ø) per hemiarch, were inserted into the jaws of five dogs, divided into two groups: chitosan-coated implant group (ChtG) and control group (CG). Twelve weeks after surgery, euthanasia was performed, and sectioned bone blocks were obtained and scanned by micro-CT and two bone parameters were measured: bone in contact with the implant surface (BCIS) and peri-implant bone area (PIBA). For BCIS and PIBA statistically significant values were obtained for the ChtG group with respect to CG (*p* = 0.005; *p* = 0.014 and *p* < 0.001 and *p* = 0.002, respectively). The results, despite the limitations, demonstrated the usefulness of chitosan coatings. However, studies with larger sample sizes and adequate experimental models would be necessary to confirm the results.

## Introduction

Dental implant treatments have now become indispensable in clinical dental practice. The survival rate exceeds 90%, although studies on success rates are difficult to interpret, mainly due to a large number of variables, such as the surgical techniques used and the follow-up periods, in addition to the different criteria that have been proposed to define implant success (Simonis et al., 2010). Modern oral im-plantology uses different devices, in terms of size, shape, length, thickness and composition, from pure titanium (Ti) to titanium-aluminum-vanadium alloys (Ti-Al-V), due to their biocompatibility and high corrosion resistance (von Wilmowsky et al., 2014). However, the biological response of tissues can be improved by different surface treatments that provide both bioactivity and osseointegration capacity (Jemat et al., 2015). The first materials used in implantology provoked marked inflammatory reactions that led to the formation of fibrous tissue around the implant, with consequent failure; however, the latest generation materials, in addition to awakening metabolic activities, do not affect the normal biological metabolism, being considered as bioinductive materials (Li et al., 2019a; Hotchkiss et al., 2019), it is currently considered that certain changes on the surface of Ti play an active role in the control of the cellular response, resulting in reduced healing times and improved healing of the peri-implant area (Le Guéhennec et al., 2007a; Alfarsi et al., 2014). Current trends are directed not only towards achieving optimal osseointegrative surfaces, but also towards surfaces with antibacterial activity for prolonged periods of time, either by blocking microbial adhesion or by preventing late infections (Palla-Rubio et al., 2019).

Chitosan (Cht) is a polysaccharide derived from partially deacetylated chitin, formed by copolymers of glucosamine and N-acetylglucosamine. It possesses several amino groups attached to the main chain of the polysaccharide, which are readily available for chemical reaction and formation of salts with acids (Singla and Chawla, 2001). In recent years, it has been proposed as a promising biomaterial in certain dental and tissue engineering applications, in addition to being used as a cholesterol-lowering agent, hemostatic, drug carrier etc. (Ylitalo et al., 2002; Rojo and Deb, 2015; Ahsan et al., 2018; Hu et al., 2018; Ahn et al., 2021; Yu et al., 2022).

Some studies consider it as bactericidal and others as bacteriostatic, although its mechanism of action in both situations is not exactly known, since different factors have been proposed as contributing to its antibacterial action, among them, the amino groups of its structure and the origin of the chitin (Rabea et al., 2003; Matica et al., 2019). Likewise, its high biocompatibility, hydrophilicity and biodegradability, in addition to being non-toxic (Tajdini et al., 2010), are noteworthy. For all these reasons, its ability to increase cell adhesion and protein adsorption in Ti coatings has been highlighted, which would be beneficial for improving the osseointegration of dental implants (Bumgardner et al., 20032003; Bumgardner et al., 2003; López-Valverde et al., 2021). Muzzarelli et al. (Muzzarelli et al., 1994) demonstrated in a clinical trial on 10 patients, bone neoformation and mineralization of post-extraction sockets, due to the cationic nature and chelating ability of Cht; these results would highlight the potential of Cht coatings to support and facilitate osseointegration of orthopedic and craniofacial implants. Cht-based implants have been found to elicit minimal foreign body reaction, with little or no fibrous encapsulation and promote a rapid healing response (Kim et al., 2008). Most implant failures are due to poor early bone healing at the bone-implant interface (Sakka et al., 2012) and in this aspect, Cht has been proposed as a biomaterial with good bioactivity for osteogenesis (Hu et al., 2009).

However, as implant surface modifications have changed, investigations have become multifactorial in an attempt to develop detailed information on design optimization, resulting in difficulty in capturing the detailed bone response in a timely manner and with sufficient resolution by current conventional methods (Vandeweghe et al., 2013a).

The good film-forming ability of Cht allows its use in the coating of dental implants and the coated surfaces show good cell compatibility with osteoblastic and fibroblastic cells (Shukla et al., 2013a). Numerous studies of Ti coatings with Cht have been performed, with the attachment of Cht to the metal substrate being considered a challenge, either by electrophoretic deposition, layer-by-layer deposition, casting methods, spin coating and dip coating methods (Bumgardner et al., 20032003; Reddy Tiyyagura et al., 2016; Chen et al., 2017; Höhlinger et al., 2017). Dip coating of a substrate, used in our study, is a simple form of deposition, especially for small substrates, forming thin layer deposits, which can be further compacted, by heat treatment. Moreover, it is an economical way to deposit thin layers from chemical solutions, with relatively fair control over the layer thickness (Grosso, 2011). Dip coating is based on a steady flow condition, and the coating thickness is determined by the competition between viscous force, surface tension, gravity and substrate withdrawal rate (Scriven, 1988).

On the other hand, some researchers have pointed out the limitations of histomorphometry in providing quantitative and qualitative bone information, due to the dependence on slice position and possible interface damage during sample cutting and grinding procedures, in addition to relying on a small number of sections, which means a limited subset of the entire sample. All this, together with the sample preparation time, the destructive nature of the method and its cost, has led to the proposal of new evaluation techniques, such as micro computed tomography (micro-CT) analysis, which increase the performance of the evaluation, providing the same resolution capacity as conventional techniques and, above all, because they take advantage of the non-destructive nature of the specimens (Kampschulte et al., 2016; Becker et al., 2017; He et al., 2017).

In addition, micro-CT produces an improved resolution in the range approximately 1,000,000 times smaller than normal CT scanning, allowing a three-dimensional (3D) evaluation of the specimen in high resolution and providing 3D reconstructed images, to obtain a better understanding of the bone architecture, generated within the area of interest (AoI) (Szmukler-Moncler et al., 2004; Boyd et al., 2006; Peyrin et al., 2014).

Therefore, the aim of our study, was to evaluate the osseointegration and bone formation at crestal, mid and apical levels of Cht-coated Ti implants in the mandible of a canine model and to compare them with conventional implants with an etched surface (SLA type) without coating. The null hypothesis was that uncoated implants, with a conventional SLA-type etched surface, have the same osseointegration and bone formation capacity as implants coated with Cht.

## Materials and Methods

### Study Design

Forty implants (8.5 mm length x 3.5 mm Ø) were inserted in the jaws of 5 Foxhound dogs, four per hemiarch. They were randomly divided into two groups: a group of im-plants re-coated with chitosan (ChtG) and a group of control implants without coating (CG). Two bone parameters were measured around the implant, Bone in Contact to the Implant Surface (BCIS) and Peri-Implant Bone Area (PIBA) at three levels: crestal, middle and apical of each implant. The study protocol was approved on 24 July 2020 by the Ethics Committee of the Catholic University of Murcia (Spain) with code CE072004.

### Implant Surface Topography

Bioner^®^ Ti implants, grade 5 (TiAl6V4) (Sant Just Desvern, Barcelona, Spain) (CG), were etched by the proprietary Bioetch^®^ method, which provides a homogeneous macro- and microtextured macropore surface in the 15–20 µm range (Höhlinger et al., 2017) (Figures 1A,B)

**FIGURE 1:** Implant surface topography. CG surface **(A,B)**. ChtG coated implant surface **(C)**.

### Implant Surface Preparation

The chitosan coating (ChtG) was prepared according to the procedure described by Vakili et al. with slight modifications (Vakili and Asefnejad, 2020). 0.5% (w/v) chitosan was prepared in 0.5% (v/v) acidic solution by stirring the solution for 12 h on a magnetic stirrer. The film-forming solution was prepared following the procedure described by Zhang et al. with slight modifications (Zhang et al., 2019). Glycerol (0.4 g) was dispersed in 80 ml of acetic acid (1%, w/v) by stirring for at least 12 h (4°C). The prepared chitosan solution was added to the film-forming solution using a syringe pump (Infusomat^®^ Space, Braun, Barcelona, Spain), at a rate of 50 ml/h, stirring by mechanical shaker at 800 rpm. The implants were coated with Cht by immersion in the prepared solution, coating the entire implant surface. The coated implants were then dried in a drying oven with rotary drum and air blowing at 25°C for the formation of a uniform film, with a relative humidity of 50%, to avoid cracking and deformation of the coating (Figure 1C). CG implants did not receive any surface coating. Both CG and ChtG implants were sterilized by gamma irradiation. This method of sterilization in ChtG was preferred so as not to give rise to sterilization biases with GC. Other methods, such as ethylene oxide, in addition to leaving residues detrimental to health, could damage the molecular structure of the coating and its susceptibility to degradation, although the effects of sterilization on the stability of the molecular structure and the mechanical properties of the coating itself are unclear. Certain *in vitro* studies have shown that the early stages of mineralization are essentially independent of the sterilization method (Ueno et al., 2012; Türker et al., 2014).

### Surgical Protocol

The surgical procedures, supervised by a veterinary surgeon, were performed under general anesthesia, infusing Propofol^®^ (Propovet, Abbott Laboratories Ltd., Queens-borough, Kent, United Kingdom), through a catheter installed in the cephalic vein. Anesthetic maintenance was performed by means of a volatile anesthetic (Isoflurane, IsoVet 1000 mg/g^®^, Piramal Critical Care B.V. Voorschoten, NL). In addition, a local anesthetic was administered to the surgical sites (articaine 40 mg, with 1% epinephrine, Ultracain^®^, Normon, Madrid, Spain). Three premolars and the first mandibular molar (P2, P3, P4 and M1) of each animal were extracted by odontosection (Figure 2). The placement of the implants in the empty sockets (Figure 2) was determined by the randomization program (http://www.randomization.com). The experimental animals were assigned to the two different implant surfaces: 20 implants with Cht from the test group (ChtG) and 20 uncoated implants from the commercial company Bioner (Bioetch^®^, Bioner Sistemas Implantológicos, Barcelona, Spain) (CG), randomly distributed among five dogs. Each dog received eight screw implants (8.5 mm length x 3.5 mm Ø in the premolar and molar area), four per hemiarch. Cover screws were placed to allow a submerged healing protocol (Figure 2). The implants were placed in the post-extraction sockets without friction of the implant with the alveolar walls (Figure 2), achieving primary stability of the implants in the apical area, so as not to damage the coating with the insertion forces, leaving the cylindrical part of the implant in contact with the blood clot and only the conical apical part in contact with the bone. Healing abutments were not placed to avoid bacterial contamination and contact with the antagonist teeth during chewing and to avoid disturbing the rest period of the implants. No grafting materials were used in the spaces between the alveolar walls and the placed implants (Figure 2). The flaps were closed with simple sutures (Silk 4-0^®^, Lorca Marín, Lorca, Spain). The animals were maintained on a soft diet from the time of surgery until the end of the study. Sacrifice was performed after 12 weeks, using pentothal natrium (Abbot Laboratories, Madrid, Spain) perfused through the carotid artery, after anesthesia of the animal. Sectioned bone blocks were obtained.

**FIGURE 2:** Surgery. **(A)**, Odontosection; **(B)**, Implant insertion; **(C)**, Implant placed in subcrestal position with cover screws for submerged curing; **(D)**, Lack of friction between the implant and the bone wall.

### Micro-Computed Tomography Analysis

After euthanasia of animals (after 12 weeks of implants placement), the sections of the block were preserved and fixed in 10% neutral formalin. Image acquisitions were per-formed using a multimodal SPECT/CT Albira II ARS scanner (Bruker^®^ Corporation, Karksruhe, Germany). The acquisition parameters were 45 kV, 0.2 mA, and 0.05 mm voxels. The acquisition slices were axial, 0.05 mm thick, and 800 to 1,000 images were obtained from each piece through a flat panel digital detector with 2,400 × 2,400 pixels and a FOV (field of view) of 70 mm × 70 mm. The implants were grouped according to the three axes (transverse, coronal, and sagittal). The sagital axis was used for BCIS and PIBA measurements. In all images the same color scale was used (0 min and 3 max) with the same parameters in FOV (%): 90 and zoom 0.6, with a hardness of 1. The areas of interest (AoIs) were manually fixed by three micro-CT cross-sections at crestal, mid and apical levels; the apical section avoided the conical area of the implant (Figure 3). The voxels in contact with the implant surface were excluded in the measurements because they were considered artifact zones, estimating a value of 0.5 mm higher than the implant diameter for the calculation of the BCIS AoI (4 mm Ø) and 2 mm for the calculation of the PIBA AoI (5.5 mm Ø) (Figure 4).

**FIGURE 3:** Areas of interest (AoI) delimited by three micro-CT slices at crestal, mid and apical level.

**FIGURE 4:** Artifact area in white color; bone in contact with the implant surface (BCIS) in green color and peri-implant bone area (PIBA) in yellow color.

The AMIDE tool allowed us to obtain the data in statistical form (Hounsfield Units), with maximums, minimums and deviations. AMIDE is a tool for visualizing, analyzing and registering volumetric medical image data sets (AMIDE, UCLA University, Los Angeles, CA, USA). It allows drawing two-dimensional and three-dimensional AoIs directly on the images and generating statistical data for these AoIs. 3D Slicer program (http://www.slicer.org) provided the 3D images of the bone-to-implant contact area (Figure 5).

**FIGURE 5:** **(A)**, Micro-CT image in sagittal plane and graph to represent the artifact area, bone in contact with the implant surface (BCIS) (4 mm Ø) and peri-implant bone area (PIBA) (5.5 mm Ø); **(B)**, 3D image with the contact and non-contact surfaces of the bone with the implant.

### Statistical Analysis

SPSS Statistics 26.0 (IBM, Chicago, IL, USA) was used as the statistical analysis program. Statistical analysis of the BCIS and PIBA variables in the crestal, mid and apical areas was performed for the experimental and control groups. The normality of the data generated by the microtomographic analyses was examined using the Shapiro-Wilk test. The mean and standard deviation of each group were proposed; the *p*-value and p for trend derived from the differences and changes in each group were presented, with a significance level of ≤0.05.

## Results

All the implants used in the 5 dogs achieved osseointegration. Two parameters, Bone in Contact to the Implant Surface (BCIS) and Peri-Implant Bone Area (PIBA) were measured in crestal, mid and apical, resulting in a total of 120 sites for each measurement parameter, in the experimental group (ChtG) and in the control group (CG).

The mean value and standard deviation of the trends for each group are shown in Tables 1, 2. For BCIS the values in crestal, mid and apical, in the experimental group (ChtG), were 3,770.11 ± 245.60, 3,245.25 ± 1,477.08 and 4,196.82 ± 453.03, respectively and 3,829.29 ± 249.08, 3,958.75 ± 1,477.08 and 4,112.13 ± 112.6, respectively, in the control group (CG). Trend analysis in the experimental group showed a higher statistical significance (*p* = 0.005) with respect to the control group (*p* = 0.014). For PIBA the values in crestal, mid and apical, in the experimental group, were 3,613.00 ± 1,109.12, 3,905.75 ± 809.65 and 3,759.17 ± 944.73, respectively and 4,162.50 ± 618.02, 3,705.20 ± 1,045.86 and 3,832.71 ± 1,201.43, respectively, in the control group. Trend analysis in the experimental group showed considerable statistical significance (*p* < 0.001) versus the control group (*p* = 0.02). Figures 6, 7 represents the boxplots of the results.

**TABLE 1:** Specific crestal, mid and apical trends in the experimental and control groups for BCIS (mean ± deviation).

BCIS	Crestal	Mid	Apical	*p-*values
ChtG	3,770.11 ± 245.60	3,245.25 ± 1,477.08	4,196.82 ± 453.03	0.005 *
CG	3,829.29 ± 249.08	3,958.75 ± 1,477.08	4,112.13 ± 112.6	0.014

BCIS, bone in contact to the implant surface; ChtG, chitosan group; CG, Control Group. General linear model (*p* ≤ 0.05). * Statistical significance.

**TABLE 2:** Specific crestal, mid and apical trends in the experimental and control groups for PIBA (mean ± deviation).

PIBA	Crestal	Mid	Apical	*p-*values
ChtG	3,613.00 ± 1,109.12	3,905.75 ± 809.65	3,759.17 ± 944.73	<0.001 *
CG	4,162.50 ± 618.02	3,705.20 ± 1,045.86	3,832.71 ± 1,201.43	0.02

PIBA*,* Peri-Implant Bone Area; ChtG, chitosan group; CG, control group. General linear model (*p* ≤ 0.05). * Statistical significance.

**FIGURE 6:** Boxplot of peri-implant bone area (PIBA) values at crestal, mid and apical levels.

**FIGURE 7:** Boxplot of bone in contact with the implant surface (BCIS) values at crestal, mid and apical levels.

## Discussion

Since Brånemark published his first study on the osseointegration of Ti implants in 1969, there have been numerous variations of their surfaces, all with the aim of achieving early and more durable osseointegration. The topography and roughness of the surfaces have been questioned in terms of osteoblastic cell differentiation and it has been shown that the attachment of this type of cells is greater on smooth surfaces, although rougher surfaces have been associated with greater cell differentiation (Bachle and Kohal, 2004; Esposito et al., 2005). Apart from surface characteristics, it is also known that osseointegration is affected by factors such as the biological compatibility of an implant (Annunziata and Guida, 2015). Therefore, to improve the bioactivity of implants, the surface can be modified by incorporating organic and inorganic phases either within or on the Ti oxide layer, using ions, inorganic molecules or organic molecules (Jiang et al., 2014; Anitua et al., 2015).

The evaluation of bone-implant contact provides evidence of an implant anchored in the bone and has traditionally been established as the most common method of evaluation, however, the concept of osseointegration has undergone variations and is now considered as “a reaction to a foreign body in which interfacial bone is formed as a defensive reaction to protect the implant from the tissues” (Albrektsson et al., 2017; Albrektsson and Wennerberg, 2019). The amount of bone in contact with the implant, as well as the frictional properties at the contact interface, are important parameters influencing bone-implant mechanics. However, the stability of implants in trabecular bone has been little studied and considering the reduced contact surface between trabecular bone and implant, it has been suggested that macroscopic phenomena such as trabeculae-implant mechanical fixation would dominate over the microscopic aspects such as friction (Huang et al., 2008; Wirth et al., 2010).

In the present study, a model was designed in the canine mandible, where 2 bone parameters were measured in the area surrounding the implant, Bone in Contact with the Implant Surface (BCIS) and Peri-implant Bone Area (PIBA), at crestal, mid and apical levels, both in the Cht-coated implant group (ChtG) and in the control group (CG), with conventional etched surface, and the results were analyzed by means of micro-CT.

Although no single animal species meets all the requirements of an ideal model, an understanding of the differences in bone architecture and remodeling between different species of experimental animals could help to select a suitable species. Most studies resort to modified and inadequate experimental models, both the experimental animal (rabbit rat...) and the implantation site, with extraoral surgical approaches (tibia, femur...), so that the results cannot be extrapolated to humans, among other reasons, because of the lack of cortical remodeling and the fact that the cessation of growth occurs much later in these species than in other mammals (Ferguson et al., 2018). On the other hand, *in vitro* cultures maintain tissues or organs without vascularization, limiting the supply of nutrients, oxygen and waste elimination and, therefore, the extrapolation of the results to the *in vivo* situation limits the model. All this, without taking into account the reduced lifespan of the cultured cells (Pizzoferrato et al., 1994). Our preclinical study used the mandible of a canine model, with greater similarity to the human in terms of bone architecture and remodeling. The dog, along with the pig, are considered valuable models for the study of tissues adjacent to dental implants, and large-breed dogs can support human dental implants (Pearce et al., 2007). To our knowledge, this is the first time that this experimental model has been used for the study of the effectiveness of Cht as a coating for dental implants.

Cht is a macromolecule that has achieved great attention in the biomedical industry, arousing great interest in bone regeneration (De Jonge et al., 2008; Ebhodaghe, 2021). It has the ability to stimulate the recruitment and adhesion of osteogenic progenitor cells, facilitating bone formation. In addition, it has been shown that no inflammatory or allergic reactions occur after topical application (Kim et al., 2003; Waibel et al., 2011; Azuma et al., 2015; Sukpaita et al., 2021).

Typically, toxic reagents, such as 3-isocyanatopropyltriethoxysilane and glutaraldehyde, are used to form Cht coatings for silanization and attachment to the Ti substrate but these techniques involve complex processing that hinders coating deposition and limits clinical applicability (Yuan et al., 2008). However, although efforts have been made to increase the bond strength of hydroxyapatite coatings on implant alloys, as they are brittle materials, it is unclear whether these high bond strengths would be necessary for the polymeric Cht material (Bumgardner et al., 2007).

The dip coating used in our study (Vakili and Asefnejad, 2020), in addition to resisting the forces used during implantation, because of the surgical technique employed, is an inexpensive way of depositing thin layers from chemical solutions, with relatively fair control over the thickness of the layer and offers the possibility of fine-tuning the amount of material that can be deposited and, therefore, the thickness of the final film. For these reasons, it is becoming increasingly popular not only in research and development laboratories, but also in industrial production. Grosso have proposed the immersion technique as a very suitable method to impregnate porosities, make nanocomposites or perform nanofusion. (Grosso, 2011); Brinker et al. (Brinker et al., 1992) pointed out wet methods, as suitable, since they are homogeneously organized in the final film, with adequate thickness control.

The amount of Cht can be adjusted by controlling the concentration of the Cht solution and certain authors have indicated that, as the amount of loaded Cht increases, its antibacterial properties increase; therefore, controlling the amount of loaded Cht would endow the Ti implant with better biological and anti-bacterial properties. Cht loading in 0.5% acidic solution, was considered adequate (Vakili and Asefnejad, 2020), although the optimization of the amount of loaded Cht, degradation rate and antibacterial effect still need to be further investigated (Li et al., 2019b). Most of the existing studies on the efficacy of Cht as a Ti coating, as we have noted above, are *in vitro* studies or *in vivo* studies on inadequate models, or that resort to complicated coating methods, or toxic products, which hinder or impair their clinical applicability (Bumgardner et al., 2007; Kung et al., 2011; Takanche et al., 2018a; Zhang et al., 2020).

Sukpaita et al. (Sukpaita et al., 2019) demonstrated the ability of Cht scaffolds to self-promote bone tissue and repair calvarial bone defects in mice. Tian et al. (Tian et al., 2014), in an *in vitro* study, indicated that Cht film loaded on a Ti surface would promote osteoblast proliferation and differentiation in a dose-dependent manner, which could represent a new approach in the treatment of Ti implants. Zhang et al. (Li et al., 2019b) showed that porous Ti with a Cht/Hydroxyapatite coating could promote osteoblast-like cell proliferation and differentiation and osseointegration *in vivo*. Bumgardner et al. (Bumgardner et al., 2007) evaluated the ability of Cht coatings on Ti to promote bone formation and osseointegration compared to calcium phosphate coatings and uncoated Ti, in a 12-weeks rabbit model, maintaining the hypothesis that it may not be important that the Cht coating persists long-term, once a good bone-implant interface has been established, in the same way that some investigators have speculated with calcium phosphate coatings (Yang et al., 2005).

Even heterotopic (extraskeletal) bone formation induced by Cht-collagen-coated Ti implants has been demonstrated *in vivo* (Kung et al., 2011). Overall, researchers conclude that Cht significantly accelerates the bone regeneration process and, therefore, in terms of its biocompatibility and osteoinductivity, it can be considered as a biomaterial of great relevance in human bone healing (Ge et al., 2004; Pang et al., 2005; Guzmán-Morales et al., 2009; Muzzarelli, 2009; Ezoddini-Ardakani et al., 2012; Mututuvari et al., 2013), which is consistent with the results obtained in our research.

The good film-forming ability of Cht allows its use in the coating of dental or orthopedic implants, and the coated surfaces have been shown to possess good cellular compatibility with fibroblast cells. Klokkevold et al. (Klokkevold et al., 1996) reported that chitosan films enhanced osteoprogenitor cell differentiation, facilitated bone formation, and inhibited fibroblast proliferation. Moreover, the activity of Cht against bacteria such as *Escherichia coli*, *Streptococcus* mutans, *Staphylococcus aureus*, *Bacillus* subtilis and *Actinomyces* naeslundii (Renoud et al., 2012; Lin et al., 2021) and to prevent oxidative damage caused by free radicals (Ngo et al., 2011) has also been demonstrated. Takanche et al. in an *in vivo* study on osteoporotic rat jaws demonstrated, by micro-CT, that Cht-coated Ti implants increased the volume and density of newly formed bone and implant osseointegration, as well as the upregulation of bone morphogenetic protein, by inhibiting osteoclastogenesis. All these and other demonstrated properties make this biopolymer a good biocompatible and bioactive osteoconductor and a useful coating for orthopedic and craniofacial implant devices.

However, in the future, it will be necessary to determine the bond strength of the coatings and changes in bond strength over time and to evaluate the degradation of the coating in lysozyme solutions in the oral environment, as degradation rates may be different in the presence of this enzyme and changes in degradation would be important for the development of the implant-tissue interface (Yuan et al., 2008). It will also be necessary to determine whether changes in initial cell growth, or differences in Cht degradation, result in less cell mineralization. In addition, it will need to be determined whether surface morphology, roughness, and coating chemistry could be related to cell and tissue responses.

In our study, two bone parameters in the vicinity of the im-plant (BCIS and PIBA) were measured by micro-CT. The best statistical significance was obtained for PIBA, in the experimental group (ChtG) (*p* < 0.001), despite the fact that all the inserted implants obtained optimal osseointegration. The maximum value was obtained for PIBA at the crestal level of M1 in ChG (6,347.05 ± 413.2) and the minimum for BCIS at the mid-level of P2 in CG (1765.03 ± 358.01).

Micro-CT currently allows observation of bone tissue in a three-dimensional manner, as well as quantitative analysis in several sections, which is not possible by histomorphometric analysis. It detects only mineralized tissue and is therefore suitable for analyzing the bony annulus and assessing bone formation around implants during healing periods; moreover, histological studies could not be performed in clinical trials (Vandeweghe et al., 2013b; Nakahara et al., 2019). Rebaudi et al. (Rebaudi et al., 2004), have proposed it as a suitable technique for the analysis of peri-implant bone tissues, proposing it as a non-destructive evaluation, which allows the analysis of the bone-implant interface. Lyu and Lee (Lyu and Lee, 2021), in a study on rabbit tibiae, reported that the measurement of bone in contact with the implant by micro-CT is feasible to evaluate implant osseointegration, obtaining results similar to histomorphometric ones, although they recognize that the method needs further optimization. Likewise, they recognize that, in most cases, they can only use one or two histological sections per implant for histomorphometric evaluation, which could lead to an over- or underestimation of the peri-implant bone.

Nevertheless, we are aware of our limitations, in terms of small sample size and difficulty in accurately detecting the bone in close contact with the implant surface, due to the thin layer of noise in the surrounding area and the microtomography settings. and the difficulty of accurately detecting the bone in close contact with the implant surface, due to the thin layer of noise in the surrounding area and the microtomography settings. These drawbacks should be taken into account when interpreting the results. In future ongoing studies, the samples will be studied by histomorphometric analysis to compare the results.

## Conclusion

The results of this preliminary study demonstrated the usefulness of Cht coatings on Ti surfaces to improve the osseointegration of dental implants. In addition, within the limitations, the use of nondestructive micro-CT analysis, seems to be useful to evaluate bone healing in the surroundings of the implant surfaces.

Since the design of the present study allowed only a preliminary analysis, the data obtained could serve as a basis for the design of future studies.

## Data Availability

The original contributions presented in the study are included in the article/Supplementary Material, further inquiries can be directed to the corresponding author.
